The article "Spiral Computed Tomography Imaging Analysis of Positioning of Lumbar Spinal Nerve Anesthesia under the Concept of Enhanced Recovery after Surgery" was published in 2022. Journal: Contrast Media Mol Imaging.

# Spiral Computed Tomography Imaging Analysis of Positioning of Lumbar Spinal Nerve Anesthesia under the Concept of Enhanced Recovery after Surgery

**DOI:** 10.1155/2022/1703250

**Published:** 2022-06-03

**Authors:** Xue Feng, Binbin Zhao, Yongqiang Wang

**Affiliations:** ^1^Department of Anesthesia Surgery, First Affiliated Hospital,Heilongjiang University of Traditional Chinese Medicine, Harbin 150040, Heilongjiang, China; ^2^Department of Outpatient, Harbin Red Cross Central Hospital, Harbin 150076, Heilongjiang, China

## Abstract

The objective of this research was to explore the effect of perioperative anesthesia management for patients based on the concept of enhanced recovery after surgery (ERAS) and the application value of the computed tomography (CT) localization method in lumbar spinal nerve anesthesia, reducing the damage caused by anesthesia. One hundred and twenty patients who underwent the lumbar spinal anesthesia in lower limb surgery were selected as the research subjects. According to puncture positioning and nursing intention, the patients were classified into the control group with 30 patients (method of anatomical landmarks), CT group with 50 patients (the CT localization), and ERAS group with 40 patients (the CT localization and the ERAS management). The effects of the anesthesia positioning method and the ERAS management were compared and analyzed. The results showed that *d* (0.32) and *r* (0.27) of exponential filtering function were notably smaller than those of R-L filtering function (*d* = 0.40, *r* = 0.39) and of S-R filtering function (*d* = 0.37, *r* = 0.36) (*P* < 0.05). Puncture time ((9.23 ± 0.32) min vs. (13.11 ± 0.45) min), puncture direction change (20% vs. 33.33%), abnormal puncture sensation (22% vs. 40%), and nerve root touch (4% vs. 23.33%) in the CT group were all lower than those in the control group. The proportion of Degree I anesthesia effect (94%) of the CT group was greatly higher than that of the control group (76.67%) (*P* < 0.05). The VAS score, time of activity and gastrointestinal function recovery, and the incidence of adverse reactions (2.5% vs. 28%) in the ERAS group were lower than those in the CT group (*P* < 0.05). All in all, the CT localization method can improve the difficulty of anesthesia puncture and improve the anesthetic effect; the ERAS nursing concept can improve the postoperative pain of patients and contribute to the prognosis of patients and have a good clinical value.

## 1. Introduction

Intraspinal anesthesia (lumbar spinal nerve anesthesia) is a kind of local anesthesia, which is currently very common in clinic. According to the different injection positions, it can be divided into epidural anesthesia, combined spinal epidural anesthesia, and subarachnoid anesthesia (also known as spinal anesthesia/lumbar anesthesia) [1–3]. Lumbar spinal nerve anesthesia is widely used in cesarean section, lower limb surgery, hemorrhoidectomy, and the supplementary treatment of cardiovascular diseases [4, 5]. The positioning of lumbar spinal nerve anesthesia has always been the focus of clinical attention because the correct lumbar space positioning is crucial to ensure the effect of anesthesia and reduce nerve injury. Currently, the method of anatomical landmarks is often used clinically. However, this method is highly dependent on patients' bony landmarks on the body surface, so it is difficult to apply it to patients with obesity or spinal/spinous deformity [6]. Hence, the method of imaging localization becomes another common method of lumbar positioning [7]. In addition, surgery usually brings great trauma and perioperative risk to patients, so the enhanced recovery after surgery (ERAS) is designed to reduce the perioperative stress and trauma [8]. ERAS is an integration of multidisciplinary interventions based on the theories of anesthesiology, surgical methods, and pain control. The ERAS concept is proposed in the joint surgery department and is successfully implemented in some gastrointestinal procedures. At present, the ERAS concept is applied for perioperative anesthesia management, with some good adoption results [9, 10].

The article "Spiral Computed Tomography Imaging Analysis of Positioning of Lumbar Spinal Nerve Anesthesia under the Concept of Enhanced Recovery after Surgery" was published in 2022. Journal: Contrast Media Mol Imaging.

Computed tomography (CT) localization has a clear imaging, which can not only evaluate the puncture plane but also show the malformation of the spine, so it helps facilitate the customization of the puncture path and improve safety [11]. Nevertheless, due to the existence of ionizing radiation, the clinical adoption of CT localization is limited to a certain extent [12]. Clinically, the low-dose CT can reduce the radiation of the conventional CT scans to 1/6–1/4 of the original, but the image quality is affected. Presently, image reconstruction by algorithms is a common method to improve the low-dose CT images, and the typical algorithm is the filtered back projection (FBP) algorithm [13]. However, when the FBP algorithm is used to reconstruct CT images, it is relatively important to select the filtering function, because an appropriate function has a vital impact on the reconstruction results and speed. The exponential filtering function can retain the characteristics of the image well [14], and it has a good adoption effect.

In summary, patients who needed lumbar spinal nerve anesthesia were selected as research subjects. The accuracy of CT localization method was evaluated by using low-dose CT scanning for puncture positioning. Moreover, the ERAS concept was used for perioperative anesthesia management of patients, and its clinical application value was analyzed to provide better effect for patients, reduce the damage caused by anesthesia, and improve the quality of life of patients.

The article "Spiral Computed Tomography Imaging Analysis of Positioning of Lumbar Spinal Nerve Anesthesia under the Concept of Enhanced Recovery after Surgery" was published in 2022. Journal: Contrast Media Mol Imaging.

## 2. Methods

### 2.1. Research Subjects

One hundred and twenty patients who received lower limb surgery in the hospital from March 2019 to March 2021 with the need for lumbar spinal nerve anesthesia were selected as the research subjects. There were 78 male patients and 42 female patients, who ranged in age from 30 to 56 years old, with an average age of (46.23 ± 12.11) years old. Their weight ranged from 45 kg to 80 kg, with an average weight of (61.11 ± 26.85) kg. Patients were classified into the control group, CT group, and ERAS group by consulting their anesthesia puncture positioning and nursing intention. In the control group, 30 patients received anesthesia puncture positioning by the conventional method of anatomical landmarks. In the CT group, 50 patients received CT scanning for puncture positioning. Besides, 40 patients in the ERAS group underwent perioperative anesthesia management with the CT localization combined with the ERAS concept. The adoption effects of the two anesthesia positioning methods in the control group and the CT group were compared and analyzed. The effects of the ERAS concept on perioperative anesthesia management for patients' postoperative recovery in the CT group and the ERAS group were compared and analyzed. This study had been approved by ethics committee of the hospital, and the patients and their families understand the situation of the study and sign the informed consent forms.

The inclusion criteria were as follows. (i) Patients who could receive the surgery under lumbar spinal nerve anesthesia through the evaluation of examination. (ii) Patients without the contraindications to anesthesia. (iii) Patients with age over 25 years old. (iv) Patients who signed the informed consent.

The exclusion criteria were as follows. (i) Patients with the resistance to anesthesia. (ii) Patients with other serious diseases, such as dysfunction of heart, liver, and kidney, blood diseases, and tumor diseases. (iii) Patients who did not complete the full experiment. (iv) Patients in pregnancy.

### 2.2. Reconstruction Algorithm of Low Dose CT

#### 2.2.1. FBP Algorithm

The “filtered” in the FBP algorithm refers to the data correction of CT image back-projection reconstruction. The simple back-projection reconstruction algorithm produces “star-like” artifacts, resulting in the decrease of CT image quality and the unclear display after reconstruction. The specific steps of the FBP algorithm are as follows.

The article "Spiral Computed Tomography Imaging Analysis of Positioning of Lumbar Spinal Nerve Anesthesia under the Concept of Enhanced Recovery after Surgery" was published in 2022. Journal: Contrast Media Mol Imaging.

First, the one-dimensional Fourier method is used to transform the projected data (at a certain angle) *q*. The transformed data are denoted as *Q*(*ω*).

(1) $$\begin{array}{c} Q\left(\omega \right)=q\cdot w^{-j2\omega }dt\left(\infty ,-\infty \right). \end{array}$$

In (1), *w* represents the projection angle and *ω* represents the Fourier coefficient.

Second, the one-dimensional weight factor *β* and *Q*(*ω*) are multiplied, and (2) is obtained.

(2) $$\begin{array}{c} Q\left(\omega \right)•\beta =q•w^{-j2\omega }\times \beta dt\left(\infty ,-\infty \right). \end{array}$$

Then, (3) shows that after the one-dimensional Fourier transform of *Q*(*ω*)•*β*, *R*(*ω*•*β*) is obtained.

(3) $$\begin{array}{c} R\left(\omega •\beta \right)=Q\left(\omega \right)\times E\left(\omega \right)\beta w^{-j2\omega }\left(\infty ,-\infty \right). \end{array}$$

Finally, in (4), all the modified functions *R*(*ω*•*β*) of 0°–180° are back-projected, and the fault image *F*(*x*, *y*) is obtained.

(4) $$\begin{array}{c} F\left(x,y\right)=\left\{\begin{array}{c} \int_{0}^{180}R\left(\omega •\beta \right)dw,\\ ↓,\\ \int_{0}^{180}R\left(\omega •\beta \right)\left(x\text{ cos }w+y\text{ sin }w\right)dw. \end{array}\right) \end{array}$$

#### 2.2.2. Filter

The effect of the filter has a direct influence on the image quality after the reconstruction. Accordingly, the quality of the filter is closely related to the choice of the filter function. The principle of the filtering function is selecting a window function *W*(*β*). Currently, the R-L filter and S-L filter are pervasive.

(5) and (6) show the filtering function of the R-L filter.

(5) $$\begin{array}{c} F_{R-L}\left(\beta \right)=\left\{\begin{array}{c} \left|\beta \right|W\left(\beta \right),\\ ⇓,\\ \left|\beta \right|rect\left(\beta /2U\right), \end{array}\right) \end{array}$$

(6) $$\begin{array}{c} \text{rect}\left(\beta /2U\right)=\left\{\begin{array}{c} 1\in \left|\beta \right|<U=1/2d,\\ 0\in \text{others.} \end{array}\right) \end{array}$$

(7) shows the filtering function of the S-L filter.

(7) $$\begin{array}{c} F_{S-L}\left(\beta \right)=1/2\left[{\left(4U/180\right)}^{2}\left(\frac{1-4U\text{sin}360U}{1-{\left(4U\right)}^{2}}\right)\right]. \end{array}$$

In equations (5)–(7), *U* represents the projection angle. Both the R-l filter and S-L filter have certain defects. For instance, the former produces an obvious Gibbs phenomenon [15], and the latter has a poor quality of low-frequency image reconstruction. Hence, the exponential window function is proposed as a filtering function to study, and its expression is shown in (8) and (9).

(8) $$\begin{array}{c} W\left(\beta \right)=e^{-a\left|\beta /2U\right|},\left|\beta \right|<U, \end{array}$$

(9) $$\begin{array}{c} W\left(\beta \right)=0,\left|\beta \right|\geq U. \end{array}$$

In (8) and (9), *e* expresses the constant and *a* expresses the parameter. When the value of *a* is different, the obtained filtering function is different. When *a*=0, *F*_*R*−*L*_(*β*) can be obtained. When *a*=0.64, the results are close to *F*_*S*−*L*_(*β*). Consequently, the exponential window function has the characteristics of R-L, S-L, and other filtering functions.

The article "Spiral Computed Tomography Imaging Analysis of Positioning of Lumbar Spinal Nerve Anesthesia under the Concept of Enhanced Recovery after Surgery" was published in 2022. Journal: Contrast Media Mol Imaging.

#### 2.2.3. Image Evaluation Index

Normalized mean square distance (*d*) and normalized mean absolute distance (*r*) were used to evaluate the effect of reconstructed images guided by the three filtering functions.

Equ. (10) shows the expression of the normalized mean square distance (*d*).

(10) $$\begin{array}{c} d={\left[\frac{\sum_{i=1}^{N}\sum_{j=1}^{M}{\left(m_{ij}-r_{ij}\right)}^{2}}{\sum_{i=1}^{N}\sum_{j=1}^{M}{\left(m_{ij}-\bar{m}\right)}^{2}}\right]}^{1/2}. \end{array}$$

Equ. (11) shows the expression of the normalized mean absolute distance (*r*).

(11) $$\begin{array}{c} r=\left[\frac{\sum_{i=1}^{N}\sum_{j=1}^{M}\left|m_{ij}-r_{ij}\right|}{\sum_{i=1}^{N}\sum_{j=1}^{M}\left|m_{ij}\right|}\right]. \end{array}$$

In (10) and (11), *i* expresses the rows in the image, *j* expresses the columns in the image, *m* expresses the pixel density of the object model, *r* expresses the pixel density of the reconstructed image, $\bar{m}$ expresses the mean density of the object model, and *N∗M* expresses the image pixels. The larger the values of *d* and *r* were, the larger the error between the reconstructed image and the original object model image was.

### 2.3. Anesthesia Positioning and Puncture

The method of anatomical landmarks was selected according to the basic situation of patients. The soft tissue depression positioning method was suitable for obese people. The C_7_ positioning method was suitable for patients without spinal deformity, and the compound anatomic marker positioning method was suitable for patients with spinal abnormalities.

For the CT localization, the 64-slice spiral CT scanner was employed for examination. The patient was placed in the conventional supine position with both knees flexed in the right position. The scanning parameters included tube voltage 120 kV, tube current 200 mA, layer thickness 3–5 mm, and screw pitch 1 : 1. The scanning sites were from the third lumbar vertebra (L3) to the first sacral vertebra (S1). The puncture position and the angle and route of the needle insertion were determined by the CT images.

For the puncture, the anesthesia puncture kit combined lumbar and epidural puncture kit (disposable, model) was used, whose specifications were AS-E/SII, and the registered standard of the medical device of the People's Republic of China was 20153660652. Besides, the epidural puncture needle (1.6 mm × 80 mm) was used as well as the lumbar anesthesia puncture needle (0.5 mm × 113 mm).

The article "Spiral Computed Tomography Imaging Analysis of Positioning of Lumbar Spinal Nerve Anesthesia under the Concept of Enhanced Recovery after Surgery" was published in 2022. Journal: Contrast Media Mol Imaging.

### 2.4. Anesthesia Management under the ERAS Concept

The patients' psychophysiological status was concerned before the surgery. Psychological counseling was performed on the patients with psychological conditions to prevent the occurrence of psychological stress. Patients were constantly reminded to abstain from drinking and fasting. If the patient had constipation, the defecation was induced within 1-2 hours before surgery. An empty stomach was maintained from 8 hours before anesthesia, and water was forbidden from 6 hours before anesthesia. If there were patients with poor gastrointestinal function, the bladder was guided to be empty to prevent postoperative hypoglycemia or vomiting.

After the surgery, the patient's position was noticed. The patient needed to keep the supine position for 6–8 hours to reduce the pressure of the spinal cord cavity, reduce cerebrospinal fluid leakage, and avoid the occurrence of headache after lumbar anesthesia. For the diet notice, cotton swabs were used to moisten the patient's lips to relieve thirst. After 6 hours, liquid food in small amounts was allowed, and it was gradually increased to the normal. The recovery conditions of consciousness, complexion, respiration, and lower limbs' muscle strength were observed. The pain degree of patients was assessed, according to which the different methods of analgesia were given. If the degree of pain was mild, the method of distracting attention was implemented. If it was severe, painkillers were taken under the doctor's advice or a pain relief pump could be used.

### 2.5. Observation Indexes

The time required for anesthesia puncture, the number of cases of puncture direction change, puncture sensation, nerve root contact, and the anesthesia effect were all observed in the control group and the CT group. The anesthetic effect was evaluated by the rating standard of clinical effect of intraspinal anesthesia (Table 1).

The recovery indexes such as the condition of out-of-bed activity and the recovery time of gastrointestinal function were recorded. The visual analog scale (VAS) scores of 2 h, 6 h, 12 h, 24 h, and 48 h after surgery were evaluated and recorded.  Figure 1 shows the scoring method. The incidence of adverse reactions, such as gastrointestinal reaction, hypoglycemia, restlessness, infection, and abnormal cardiac function in the two groups was observed.

The article "Spiral Computed Tomography Imaging Analysis of Positioning of Lumbar Spinal Nerve Anesthesia under the Concept of Enhanced Recovery after Surgery" was published in 2022. Journal: Contrast Media Mol Imaging.

### 2.6. Statistical Method

SPSS 22.0 was employed for data processing. The quantity statistics were expressed by *x* ± *s*. The *t*-test and the *χ*^2^ test were used. The percentage (%) was how the statistics of numbers were expressed. The difference was statistically significant with *P* < 0.05.

## 3. Results

### 3.1. Reconstruction Effects of Different Filtering Functions

Figure 2 shows the comparison between normalized mean square distance (*d*) and normalized mean absolute distance (*r*) of reconstructed images by the exponential filtering function, the R-L filtering function, and the S-R filtering function. Both *d* (0.32) and *r* (0.27) of the exponential filtering function were lower than those of the R-L filtering function (*d* = 0.40, *r* = 0.39) and the S-R filtering function (*d* = 0.37, *r* = 0.36) (*P* < 0.05).  Figure 3 shows the comparison of the effect images after CT image reconstruction. The reconstructed image quality guided by the exponential filtering function was remarkably better than that guided by the other two filtering functions.

### 3.2. Comparison of the General Data

Figure 4 shows the comparison of gender, age, and weight distribution of general data of patients in the three groups. There were insignificant differences in gender distribution, average age, and average weight among the three groups (*P* > 0.05), which reflected that the experiment had certain feasibility.

### 3.3. Puncture

The time required for puncture, the number of patients with puncture direction change, the abnormal puncture sensation, and the occurrence of nerve root contact in the control group and the CT group were analyzed (Figure 5). In the control group, the puncture time was (13.11 ± 0.45) min, the number of patients with puncture direction change was 10 (33.33%), 12 patients (40%) had abnormal puncture sensation, and 7 patients (23.33%) had nerve root contact. In the CT group, the puncture time was (9.23 ± 0.32) min, the number of patients with puncture direction change was 10 (20%), 11 patients (22%) had abnormal puncture sensation, and 2 patients (4%) had nerve root contact. The results showed that the puncture time, the number of patients with puncture direction change, the abnormal puncture sensation, and the occurrence of nerve root contact in the CT group were all lower than those in the control group (*P* < 0.05).

### 3.4. Anesthesia Effect

Among the 30 patients in the control group, there were 23 (76.67%) patients with the anesthesia effect of Degree I, 3 (10%) patients with that of Degree II, 3 (10%) patients with that of Degree III, and only 1 patient with that of Degree IV. Among the 50 patients in the CT group, there were 47 (94%) patients with anesthesia effect of Degree I, 3 (6%) patients with that of Degree II, 0 (0%) patient with that of Degree III, and 0 (0%) patient with that of Degree IV. According to comparison and analysis, the proportion of Degree I in the CT group was significantly higher than that in the control group (*P* < 0.05) (Figure 6).

The article "Spiral Computed Tomography Imaging Analysis of Positioning of Lumbar Spinal Nerve Anesthesia under the Concept of Enhanced Recovery after Surgery" was published in 2022. Journal: Contrast Media Mol Imaging.

### 3.5. VSA Score

In Figure 7, the VAS scores of 2 h, 6 h, 12 h, 24 h, and 48 h after surgery were compared between the CT group and the ERAS group. The VAS scores of 2 h, 6 h, 12 h, 24 h, and 48 h after surgery in the CT group were (3.01 ± 0.89), (2.77 ± 0.59), (2.65 ± 0.78), (2.21 ± 0.74), and (1.61 ± 0.72), respectively. The VAS scores of 2 h, 6 h, 12 h, 24 h, and 48 h after surgery in the ERAS group were (1.57 ± 0.66), (1.29 ± 0.45), (1.35 ± 0.28), (0.89 ± 0.64), and (0.61 ± 0.60), respectively. The VAS scores in the ERAS group were lower than those in the CT group during the whole postoperative period (*P* < 0.05).

### 3.6. Rehabilitation Index and Adverse Reactions

Among the 50 patients in the CT group, the mean activity time and the recovery time of gastrointestinal function were (39.88 ± 6.04) hours and (11.98 ± 0.44) hours, respectively. Among the 40 patients in the ERAS group, the mean activity time and gastrointestinal function recovery time were (25.14 ± 4.74) hours and (5.69 ± 0.49) hours, respectively. The required time in the ERAS group was markedly shorter than that in the CT group (*P* < 0.05). As for the adverse reactions, in the CT group, 5 (10%) patients had gastrointestinal reactions, 2 (4%) had hypoglycemia, 3 (6%) had restlessness, 2 (4%) had the infection, and 2 (4%) had an abnormal cardiac function, and the total incidence of adverse reactions was 28%. In the ERAS group, only one (2.5%) patient had gastrointestinal reactions, and nobody had hypoglycemia, restlessness, the infection, and an abnormal cardiac function, with a total incidence of 2.5%. The total incidence of the ERAS group was observably lower than that of the CT group (*P* < 0.05) (Figure 8).

## 4. Discussion

Lumbar spinal nerve anesthesia has been widely used as a common method of local anesthesia. Accurate puncture positioning and puncture path are of great significance for the reduction of anesthetic effects and adverse reactions. With the development of imaging technology, CT scanning localization has become one of the key technologies, and it is also one of the themes of the experiment.

In the experiment, there was ionizing radiation in the conventional CT examination. Consequently, the low dose CT scanning technology and the FBP algorithm were used to reconstruct CT images to prevent the degradation of the image display effect. The performance of the FBP algorithm was related to the filtering function. Furthermore, the exponential filtering function could keep the good reconstruction characteristic of the FBP algorithm [16]. The values of *d* (0.32) and *r* (0.27) of exponential filtering function were manifestly smaller than those of the R-L filtering function (*d* = 0.40, *r* = 0.39) and the S-R filtering function (*d* = 0.37, *r* = 0.36) (*P* < 0.05). The results reflected that the error between the reconstructed image and the original image of the exponential filtering function was smaller than that of both the R-L filtering function and the S-R filtering function, with the ideal reconstructed image quality, which was consistent with the above research results.

The article "Spiral Computed Tomography Imaging Analysis of Positioning of Lumbar Spinal Nerve Anesthesia under the Concept of Enhanced Recovery after Surgery" was published in 2022. Journal: Contrast Media Mol Imaging.

Based on the above results, the anesthesia puncture process and the anesthesia effect were compared between the method of anatomical landmarks and the CT localization. The incidence of puncture time (9.23 ± 0.32) min vs. (13.11 ± 0.45) min), puncture direction change (20% vs. 33.33%), abnormal puncture sensation (22% vs. 40%), and nerve root contact (4% vs. 23.33%) in the CT group were lower than those in the control group. The proportion of Degree I anesthesia effect (94%) of the CT group was signally higher than that of the control group (76.67%) (*P* < 0.05). The CT localization had a good adoption value in lumbar spinal nerve anesthesia positioning. According to many clinical investigations, the improper intraspinal anesthesia puncture brings adverse consequences to patients, while the imaging puncture positioning brings benefits to patients to a certain extent [17, 18]. The value of CT examination in lumbar spinal anesthesia is investigated. The results show that the success rate of surgery is higher in patients with the CT examination than in those without [19]. Sun et al. [20] found that imaging technology was an effective and tolerable method for the guidance of local anesthesia.

In recent years, it has been proposed that if there is no nursing intervention during the perioperative period of anesthesia, patients will often have serious physiological and psychological reactions after surgery, which are not conducive to their prognosis [21]. The ERAS concept is thus mentioned and applied to ensure the quality of nursing during the recovery of anesthesia [22]. Perioperative nursing with the ERAS concept can effectively improve patients' pain and facilitate postoperative recovery [23, 24]. Moreover, in this work, the VAS scores in the ERAS group were lower than those in the CT group at all the postoperative periods, and the time required for activity and gastrointestinal function recovery in the ERAS group was greatly shorter than that in the CT group (*P* < 0.05). Anesthesia nursing under the ERAS concept had the effect of improving patients' pain and promoting patients' postoperative recovery, which was consistent with the above research results. Besides, the total incidence of adverse reactions in the ERAS group (2.5%) was significantly lower than that in the CT group (28%) (*P* < 0.05). Mancel et al. [25] proposed that the implementation of ERAS nursing in different surgical procedures helped reduce the overall complications and the recovery time. Chiu et al. [26] proposed that ERAS nursing could improve the analgesic effect and reduce the occurrence of some adverse reactions like nausea and vomiting. Hence, the good adoption prospect of the ERAS concept in the perioperative period was reflected.

The article "Spiral Computed Tomography Imaging Analysis of Positioning of Lumbar Spinal Nerve Anesthesia under the Concept of Enhanced Recovery after Surgery" was published in 2022. Journal: Contrast Media Mol Imaging.

## 5. Conclusion

The adoption value of the CT localization in lumbar spinal nerve anesthesia positioning was analyzed under the ERAS concept, and the effect of perioperative anesthesia management under the ERAS concept was evaluated. The results proved that the CT localization was helpful to improve the difficulty of anesthesia puncture as well as the anesthesia effect. The ERAS nursing could improve postoperative pain and contribute to patients' prognosis, both of which had a favorable clinical adoption value. However, the radiation in the CT scanning used in this work cannot be eliminated at present, so the selection of research subjects is limited, resulting in an incomplete study population. This deficiency needs to be improved and broken through in subsequent explorations. The ERAS concept has good development prospects in clinical disease care, and it is worthy of further clinical exploration.

## Figures and Tables

**Figure 1:** Scoring method of VAS.

**Figure 2:** Values of (*d*) and (*r*) of different filtering functions. ^*∗*^ Compared with the exponential filtering function, *P* < 0.05.

**Figure 3:** Effect images after reconstruction.

**Figure 4:** Comparison of general data. 1: male; 2: female.

**Figure 5:** Comparison of puncture conditions. (a) Time required for puncture; (b) puncture condition (number of cases with changed direction (F), abnormal sensation of puncture (Y), and nerve root touch (P)). ^∗^ indicates that there is a statistically significant difference in the time required for puncture and the number of cases with changed direction compared with the control group (*P* < 0.05).

**Figure 6:** Comparison of anesthesia effect. ^*∗*^ Compared with CT group, *P* < 0.05.

**Figure 7:** VAS score. ^*∗*^ Compared with CT group, *P* < 0.05.

**Figure 8:** Comparisons of the rehabilitation index and the incidence of adverse reactions. (a) Activity time and (b) recovery time of gastrointestinal function. ^*∗*^ Compared with CT group in ambulation time, intestinal function recovery time, and incidence of adverse reactions, *P* < 0.05.

The article "Spiral Computed Tomography Imaging Analysis of Positioning of Lumbar Spinal Nerve Anesthesia under the Concept of Enhanced Recovery after Surgery" was published in 2022. Journal: Contrast Media Mol Imaging.

**Table 1:** Rating standard of clinical effect of intraspinal anesthesia.

Degree	Anesthesia	Pain	Muscle	Hemodynamics	Adjuvant drugs	Surgery
I	Perfect	Painless	Relaxed	Stable	Not required	Easy
II	Nearly perfect	Mild	Not good enough	Fluctuant	Required	Nearly easy
III	Imperfect	Obvious	Poor	Obvious fluctuation	Required	Fair

## Data Availability

The data used to support the findings of this study are available from the corresponding author upon request.
